The article "Contrast-Enhanced Ultrasound and Magnetic Resonance Enhancement Based on Machine Learning in Cancer Diagnosis in the Context of the Internet of Things Medical System" was retracted in 2023. Reasons: suspected computer-generated content; unreliable results or conclusions; lack of ethics approval or compliance; missing or withdrawn patient consent.

# Contrast-Enhanced Ultrasound and Magnetic Resonance Enhancement Based on Machine Learning in Cancer Diagnosis in the Context of the Internet of Things Medical System

**DOI:** 10.1155/2022/4378173

**Published:** 2022-07-14

**Authors:** Guo Zhou, Yongliang Zhang, Yijuan You, Binghua Wang, Simin Wang, Chong Yang, Yu Zhang, Jun Liu

**Affiliations:** ^1^Department of Ultrasound, Sichuan Provincial People's Hospital, University of Electronic Science and Technology of China, Chengdu, China; ^2^Chinese Academy of Sciences Sichuan Translational Medicine Research Hospital, Chengdu 610072, China; ^3^Medical Information Center, Sichuan Provincial People's Hospital, University of Electronic Science and Technology of China, Chengdu, China; ^4^Department of Hepatobiliary Surgery, Sichuan Provincial People's Hospital, University of Electronic Science and Technology of China, Chengdu, China

## Abstract

As an accurate, safe, and effective noninvasive examination method, imaging examination has been widely used in the diagnosis and differential diagnosis of focal liver lesions. Enhanced ultrasonography (CEUS), enhanced CT (CECT), and enhanced magnetic resonance imaging (CEMRI) are the most commonly used enhanced imaging methods in clinical practice, all of which can accurately determine the nature of liver lesions. The purpose of this paper is to study the application of contrast-enhanced ultrasound and magnetic resonance enhancement in cancer diagnosis based on the Internet of Things medical system. The basic clinical data, CEUS, and enhanced CT/MRI findings of 120 CHC patients were retrospectively analyzed. The clinicopathological features of CHC patients were investigated by contrast-enhanced ultrasonography and CT/MRI enhanced mode. The diagnostic value of contrast-enhanced ultrasound and enhanced CT/MRI combined with tumor markers in CHC was analyzed. The experimental results showed that the sensitivities of CEUS, enhanced MRI, and their combination in diagnosing CHC were 72.44%, 81.56%, and 93.78%, respectively. This experiment has an important value in the diagnosis of primary liver cancer.

## 1. Introduction

Primary liver cancer usually develops from cirrhotic regenerative nodules (RN) to dysplastic nodules (DN) and eventually progresses to early HCC [1]. The phenotype of RN is normal in nature and is generally considered to be benign, whereas DN has some features similar to well-differentiated HCC, such as disorganized arteries, clonal-like features, and varying degrees of cellular atypia [2]. Some DNs may contain tiny HCC nodules and even show signs of nodules within nodules. The development of HCC has a tendency to invade and metastasize, and most patients with early HCC have no symptoms, so most HCC patients have a poor prognosis [3, 4]. In addition to the changes at the cellular and histological levels, another key to the development of HCC is that it has special hemodynamic changes. During the gradual development process from cirrhosis of RN and DN to early HCC, the blood supply of portal vein and normal hepatic artery gradually decreased, while the blood supply of abnormal hepatic artery gradually increased, and finally, HCC was mainly supplied by the abnormal hepatic artery. Dynamic contrast-enhanced imaging examinations, for example, comparing CEUS and CEMRI, can very effectively reflect the hemodynamic characteristics of focal liver lesions and are used in the screening of HCC. It plays an extremely important role in monitoring, diagnosis, staging, and management [5, 6].

The article "Contrast-Enhanced Ultrasound and Magnetic Resonance Enhancement Based on Machine Learning in Cancer Diagnosis in the Context of the Internet of Things Medical System" was retracted in 2023. Reasons: suspected computer-generated content; unreliable results or conclusions; lack of ethics approval or compliance; missing or withdrawn patient consent.

Computer-aided diagnosis (CADx) systems help physicians make quick decisions in the field of medical imaging [7]. Nesamani et al. used mammography images, both normal and pathological, in the experiments. Machine learning classifiers are used to identify a given image as benign or malignant. The performance of both classifiers was recorded, and the neural network classifier was observed to perform well in diagnosis [8]. Al used Ant-Miner, a classification algorithm based on ant colony optimization, to analyze the cervical cancer data set. The proposed algorithm has better classification accuracy in the same domain [9]. Therefore, it is of practical significance to study the analysis of cancer diagnosis based on machine learning in the context of the Internet of Things medical system.

Methods: The clinical data of patients with focal liver lesions in the background of chronic liver disease were collected. The pathological results of surgical resection or needle biopsy were collected, and the accuracy of CEUS and CEMRI in diagnosing HCC was calculated using clinical diagnostic test methods. To compare the diagnostic effects of CEUS, enhanced MRI and their combined diagnosis of CHC, and to explore whether combined diagnosis can further improve the diagnostic performance.

## 2. Research on Contrast-Enhanced Ultrasound and Magnetic Resonance Enhancement Based on Machine Learning in Cancer Diagnosis in the Context of the Internet of Things Medical System

### 2.1. The Application of IoT in the Medical Field

In the medical field, the application of IoT technology in telemedicine can realize the intelligentization of medical services. Intelligent medical care can make the hospital better informatization and improve the efficiency of patients' settlement and treatment within the hospital; it can coordinate medical actions through regional medical collaboration and improve the influence of crossregional medical care [10].

The article "Contrast-Enhanced Ultrasound and Magnetic Resonance Enhancement Based on Machine Learning in Cancer Diagnosis in the Context of the Internet of Things Medical System" was retracted in 2023. Reasons: suspected computer-generated content; unreliable results or conclusions; lack of ethics approval or compliance; missing or withdrawn patient consent.

The intelligent medical information system integrates various patient information and shares it with medical staff, government administrators, patients, and other medical service providers [11]. The integration of different patient information makes the science and even the economy of medical and health services more convenient. It is mainly manifested in better access to medical data, prevention of medical errors and unnecessary duplication of examinations, cost savings, reduced waiting time, and reduced medical expenses [12].

A typical IoT architecture is divided into a conceptual layer, a network layer, and an application layer. The IoT layer includes many smart devices, including physiological parameter detectors, QR codes, readers, etc. These tracking devices are able to detect, identify objects, and collect raw information. IoT technology focuses on developing more expensive and comprehensive search tools, using state-of-the-art sensor technology to address low power consumption, miniaturization, and low cost. The IoT gateway is used to realize the interconnection of internal and external networks and is a very important IoT device. The IoT gateway is the link between the wireless sensor network and the traditional communication network. It integrates data monitoring and transmission and is used to complete the protocol conversion between different types of networks and realize the data collection and remote control of nodes. On the one hand, the network layer connects many search engines to network bearer services quickly and securely through interfaces and processes such as mobile networks and the Internet, so as to realize network connection and transmission of large amounts of search information. On the other hand, many trading systems are connected to the business layer through open and innovative interfaces, such as many key trading platforms and services that contain value. The application layer interacts with the network layer through open functional interfaces and the perception layer interacts with the network layer through interaction interfaces. The application layer focuses on processing common sense data, physiological parameter control, and alarming.

### 2.2. Machine Learning

Machine learning is an extremely important branch of the fundamental field [13]. At this stage, machine learning is divided into shallow learning and deep learning. At present, deep learning methods have become the mainstream methods in the field of medical image processing and analysis, including CT image liver and tumor segmentation. Compared with traditional machine learning algorithms, deep learning can only achieve the mapping of features to task targets and deep learning can realize feature learning., feature abstraction, feature-to-task target mapping, and other tasks to achieve end-to-end data-to-task target direct mapping [14, 15].

The article "Contrast-Enhanced Ultrasound and Magnetic Resonance Enhancement Based on Machine Learning in Cancer Diagnosis in the Context of the Internet of Things Medical System" was retracted in 2023. Reasons: suspected computer-generated content; unreliable results or conclusions; lack of ethics approval or compliance; missing or withdrawn patient consent.

The convolutional neural network is an important variant of the artificial neural network [16, 17]. Due to the characteristics of convolution operation, the convolutional neural network has obvious advantages for the analysis and recognition of grid-like structure data mainly based on images. Their physical meanings are as follows:

1. The number of convolution kernels *K*. The convolutional layer usually contains 2″ convolution kernels, which are, respectively, used to extract features from different patterns existing in the input tensor. Generally, the more the number of convolution kernels, the stronger the representation ability of the convolutional neural network. The number determines the number of channels of the output feature map tensor;
2. The spatial dimension *F* of the convolution kernel. The hyperparameter indicates the width or height of the convolution kernel. Usually, the width and height of the convolution kernel are the same, and they are both odd-numbered pixels, and the size of the convolution kernel is *F*1 × *E*1 × *C*1;
3. Convolution kernel sliding step size *S*. The sliding step size determines the movement range of the convolution kernel in the width and height of the input tensor. In order to ensure that the convolution kernel can traverse all the positions of the input tensor, the value of the sliding step size is usually set to be no greater than the spatial size of the convolution kernel.
4. The padding size *P* of the input tensor. This hyperparameter determines the width of padding zeros on the periphery of the input tensor and is usually used in conjunction with the convolution kernel spatial size *F* and the sliding step size *S* to flexibly control the spatial size of the output feature map tensor.

The feature classifier of ResNet and its later networks consists of a global average pooling layer and a point convolutional layer. Let the size of the feature map output by the feature extractor be *Wo* × *Ho* × *Co*, and the global average pooling layer is responsible for converting the feature map size to *l* × *l* × *Co*, that is, the number of channels remains unchanged and the spatial size is reduced to only unit width. The point convolution layer is responsible for nonlinear mapping of the converted feature map and converts the size of the feature map from *l* × *l* × *Co* to *l* × *l* × *N*, where *N* is the number of categories of the classification task, and finally, the SoftMax layer is activated to obtain the probability distribution of each category. The point convolution layer makes full use of the local connection characteristics of the convolution operation, which greatly reduces the trainable parameters of the feature classifier compared with the fully connected layer, which reduces the network volume and effectively avoids the occurrence of overfitting.

The article "Contrast-Enhanced Ultrasound and Magnetic Resonance Enhancement Based on Machine Learning in Cancer Diagnosis in the Context of the Internet of Things Medical System" was retracted in 2023. Reasons: suspected computer-generated content; unreliable results or conclusions; lack of ethics approval or compliance; missing or withdrawn patient consent.

### 2.3. Medical Images

#### 2.3.1. CEUS

Ordinary ultrasound has been widely used in the examination and diagnosis of liver lesions, and it is also the routine and preferred imaging method after liver transplantation. However, general ultrasound and general CT are not of high value for the qualitative diagnosis of recurrent lesions [18]. With the development of imaging technology, the methods used to evaluate the microcirculation perfusion of the lesions to help determine the benign and malignant lesions include contrast-enhanced ultrasonography and enhanced CT. Both two-dimensional ultrasound and color Doppler ultrasound cannot display low-velocity blood flow signals in lesions. CEUS can clearly display the microcirculation blood flow signals of lesions. Therefore, CEUS is regarded as the “third revolution” in the field of ultrasound [19, 20].

#### 2.3.2. MRI

Magnetic resonance imaging is a technique that uses nuclear magnetic resonance technology to capture images by reconstructing the signals produced by atomic nuclei in a magnetic field. It has the advantages of non-invasiveness and high spatial resolution. In just half a century, MRI technology has made a very rapid development, and now, it has become one of the routine imaging methods [21].

## 3. Investigation and Research of Contrast-Enhanced Ultrasound and Magnetic Resonance Enhancement Based on Machine Learning in Cancer Diagnosis in the Context of Internet of Things Medical System

### 3.1. Instruments and Methods

#### 3.1.1. Research Subjects

A retrospective analysis was performed on 120 patients who came to the Medical University for suspected HCC from January 1, 2019 to January 1, 2022, including 50 CKD patients and 50 non-CKD patients. They were aged 50 to 80 years old, with an average of 66 years old.

#### 3.1.2. Contrast-Enhanced Ultrasound

We used the Philips iU Elite or Epic ultrasound system, equipped with a convex vibration sensor C5-1, a frequency 1.0∼5.0 MHz, a mechanical index 0.06–0.08; the Siemens Acuson S3000 ultrasound system and Acuson Sequoia vi6x1, with a frequency 1.0∼6.0 MHz, a mechanical indicator 0.08–0.10, all equipped with enhanced contrast ultrasound software. The contrast agent was SonoVue.

#### 3.1.3. Enhanced MRI

Scanned with Siemens MagnetomVerio3.0T magnetic resonance apparatus, conventional rotation echo (SE) T1WI/T1WI-FS and fast rotation (FSE) T2WI/T2WI-FS and DWI were displayed. SET1WI: TR750 ms, TE12 ms, FSET2WI: TR5000 ms, TE107 ms, layer thickness 4.0 mm, matrix 320 × 256. Before the examination, it was confirmed that the patient had no contraindications to MRI. Then, we injected Gd-DTPA contrast agent 0.0025 mmol/kg, 1.0 mL/s plastic and then rinsed it with 25 mL of normal saline. Arterial, portal, and delayed phase scans were performed at 15–18, 50–60, and 180, respectively.

The article "Contrast-Enhanced Ultrasound and Magnetic Resonance Enhancement Based on Machine Learning in Cancer Diagnosis in the Context of the Internet of Things Medical System" was retracted in 2023. Reasons: suspected computer-generated content; unreliable results or conclusions; lack of ethics approval or compliance; missing or withdrawn patient consent.

### 3.2. IoT Medical System Data Transmission Layer

The design of the data transmission layer protocol mainly solves the channel of the application program to ensure the reliable transmission of the message. Among them, the reliable data transmission adopt the well-known “three-way handshake” process. The data transmission layer protocol mainly realizes the control of data transmission and the format of user data message. Therefore, the data transmission layer protocol includes transmission control frames and message frames. The type area of the data transmission control frame indicates the type of the data transmission control frame, and its values are shown in Table 1:

The data were collected and arranged by the Internet of Things medical system, and SPSS17.0 software (IBM) was used for statistical analysis. The inspection results were used as the diagnostic criteria, and *t*-test was carried out:

(1) $$\begin{array}{c} t=\frac{\bar{X}-\mu }{\sigma X/\sqrt{n}}. \end{array}$$

Among them, formula (1) is a general test, *s* is the sample standard deviation, and *n* is the number of samples.

The Pearson compatibility of version *X* and version *y* are multiplied as follows:

(2) $$\begin{array}{c} r=\frac{\sum_{i=1}^{n}\left(X_{i}-\overset{¯}{X}\right)\left(Y_{i}-\overset{¯}{Y}\right)}{\sqrt{\sum_{i=1}^{n}{\left(X_{i}-\overset{¯}{X}\right)}^{2}}\sqrt{\sum_{i=1}^{n}{\left(Y_{i}-\overset{¯}{Y}\right)}^{2}}}, \end{array}$$

where *X*_*i*_ is the sum of the *X* parts of the *i*th sample, which is the sum of the *y* parts of the *i*th sample, $\bar{X}$ is the sum of the *X* parts of all samples, and $\bar{Y}$ is the sum of the *y* parts of all samples. The absolute value of the Pearson correlation coefficient is between 0 and 1, and the larger the value, the stronger the correlation between the two features.

## 4. Analysis and Research of Contrast-Enhanced Ultrasound and Magnetic Resonance Enhancement Based on Machine Learning in Cancer Diagnosis in the Context of the Internet of Things Medical System

### 4.1. Enhanced CT/MRI Manifestations

In the IoT medical system, the VNet has 5 layers, and the size of the convolution kernel in the residual module is 5 × 5 × 5. The supervised module usually consists of several fully connected layers or convolutional layers and an auxiliary loss function to extract the intermediate feature maps of the network. During the forward propagation, the output results are obtained in advance, and the additional gradient information from the auxiliary loss function is directly injected into the network during the back propagation.

The article "Contrast-Enhanced Ultrasound and Magnetic Resonance Enhancement Based on Machine Learning in Cancer Diagnosis in the Context of the Internet of Things Medical System" was retracted in 2023. Reasons: suspected computer-generated content; unreliable results or conclusions; lack of ethics approval or compliance; missing or withdrawn patient consent.

In the CT liver and tumor segmentation tasks, the samples of the 3D dataset are segmented volume data, while the samples of the 2D dataset are slice data, so the dataset used for training the 3D network is smaller. In addition, the parameters of the 3D network are smaller. The amount of network is usually more than that of a two-dimensional network, which makes the network optimization challenge in this task more severe. Therefore, LW-VNet also introduces a deep supervision module outside the backbone network, and its structure is shown in Figure 1.

The feature map output by each level of the decoder is first adjusted by point convolution, which is used to adjust the number of channels of the intermediate feature map to the number of classification categories, and then, the feature map is upsampled to the same spatial size as the label through trilinear interpolation. Finally, the probability map of the segmentation result is obtained through the SoftMax layer calculation.

In this paper, a CT image of a research subject was randomly selected for imaging performance analysis. Plain CT and enhanced CT are shown in Figure 2.

The size of the liver was normal, the liver limbs were not smooth, the density of the liver parenchyma was unevenly reduced, and no abnormal enlargement was found. The gallbladder, spleen, pancreas, kidney, and adrenal gland were all unremarkable. No obvious abnormality was found on scan and bowel. There was no effusion in the abdominal cavity. There were no enlarged lymph nodes in the abdominal cavity and retroperitoneal space.

This paper further analyzes its magnetic resonance imaging performance: it is a fragmentary reduction of the liver signal inverse phase. The liver parenchyma was rough, and the carpal tunnel was slightly enlarged. There was no obvious dilatation and no abnormality was found in the course of intrahepatic blood vessels and intravascular signals. Nodular shadows can be seen in the lower part of the right posterior lobe. The T1 signal shadow is slightly longer, and the T2 signal shadow is slightly larger. After magnification, the annular continuous magnification is uneven. There were several small round shadows of T1 signal and long shadows of T2 in the liver, and no abnormal enlargement was found after magnification.

The article "Contrast-Enhanced Ultrasound and Magnetic Resonance Enhancement Based on Machine Learning in Cancer Diagnosis in the Context of the Internet of Things Medical System" was retracted in 2023. Reasons: suspected computer-generated content; unreliable results or conclusions; lack of ethics approval or compliance; missing or withdrawn patient consent.

### 4.2. Comparison of CEUS, Enhanced MRI, and Combined Diagnosis

The sensitivities of CEUS, enhanced MRI, and their combination in diagnosing CHC were 72.44%, 81.56%, and 93.78%, respectively, as shown in Table 2. The specificity was 75.86%, 83.73%, and 78.62%, and the accuracy was 80.21%, 89.11%, and 88.82%, respectively, as shown in Figure 3.

There was no significant difference in the sensitivity of CEUS and MRI in the diagnosis of CHC (*P* > 0.05), as shown in Figure 4. The difference in the diagnostic sensitivity of the two techniques at the same time and a single technique was statistically significant (*P* < 0.05), and the difference in the accuracy of the CEUS and the combined application of the two in the diagnosis of CHC was not statistically significant (*P* > 0.05). The results are shown in Table 3.

## 5. Conclusion

CHC is a special histopathological type of primary liver cancer. The research on the diagnostic criteria and treatment methods of CHC has always attracted people's attention. This paper first analyzes the application of IoT in the medical field and studies the convolutional neural network in machine learning. The performance of enhanced CT/MRI in the diagnosis of cancer in the Internet of Things medical system was analyzed. This study found that a small number of CHC lesions have inconsistent enhancement patterns between CEUS and contrast-enhanced CT/MRI, showing that the two are contradictory, so they were included in the diagnostic criteria for CHC. Finally, CEUS, contrast-enhanced CT/MRI and ultrasound were calculated. The diagnostic value of contrast-enhanced CT/MRI combined with contrast-enhanced CT/MRI results in the highest diagnostic sensitivity. The reason may be that some CHC lesions have typical enhancement patterns on enhanced CT/MRI, and some lesions have differences in contrast-enhanced ultrasound and enhanced CT/MRI. Sexual performance is also suggestive of CHC.

The reasons for the misdiagnosis were as follows: (1) The biological characteristics of the tumor itself led to an unclear contrast between the portal venous phase and the delayed phase. When the malignancy of the lesion increases, the proportion of blood supply to the portal vein of the lesion decreases, and new blood vessels grow rapidly, so that the arterial blood supply to the lesion first decreases and then increases. (2) The influence of the lesion site, patient position, respiratory rate, etc.; (3) Two contrast agents. The principle and characteristics of perspiration are different: the ultrasound contrast agent is a blood concentration detector, which is metabolized in the body through pulmonary respiration, and the metabolism is fast, so that some lesions cannot be clearly displayed, causing errors; while the enhanced CT contrast agent is a non-ionic contrast agent. Ioversol can overflow the blood vessels and enter the extracellular space to reduce the difference in the distribution of contrast agents inside and outside the blood vessels, resulting in errors.

The article "Contrast-Enhanced Ultrasound and Magnetic Resonance Enhancement Based on Machine Learning in Cancer Diagnosis in the Context of the Internet of Things Medical System" was retracted in 2023. Reasons: suspected computer-generated content; unreliable results or conclusions; lack of ethics approval or compliance; missing or withdrawn patient consent.

Contrast-enhanced CT can perform rapid scanning, and a full abdominal scan only requires the patient to hold one breath, and there is no scanning blind spot. In the comprehensive display of lesions, enhanced CT has unique advantages. However, for some small lesions, the contrast-enhanced CT is not good for small lesions due to the influence of slice thickness. In addition, due to the intermittent scanning imaging of contrast-enhanced CT, the diagnostic performance of some lesions is poor. Because the early symptoms of CHC patients are insidious, early diagnosis is very important.

CEUS is a continuous dynamic imaging technology with a high temporal resolution. The contrast agent used is not only well tolerated but also has no liver and kidney toxicity and has a low incidence of allergic reactions. Compared with CEMRI and CECT, it is more economical and convenient, and it acts as a pure blood pool. The contrast agent, which can always remain in the vascular lumen and will not spread to the interstitial space, is of great value in diagnosing HCC with abnormal hepatic arterial blood supply in the arterial phase. CEMRI not only has the dynamic enhancement function of blood perfusion but also has rich image acquisition signals, high soft tissue resolution, and no radioactive radiation. It can also provide clinical information such as liver metabolism and pathophysiology. CECT has a clear tissue contrast, but relatively low temporal resolution and radioactive radiation.

## Figures and Tables

**Figure 1:** LW-VNet structure.

**Figure 2:** CT image.

**Figure 3:** Comparison results.

**Figure 4:** Statistically significant results.

**Table 1:** Types and values of data transmission control frames.

Frame type	Value
Transmission request frame	0 × 01
Transmission confirmation frame	0 × 02
User data frame	0 × 03

**Table 2:** Comparison of CEUS and contrast-enhanced MRI and combined diagnostic sensitivity, specificity, and accuracy.

Index	CEUS (%)	Enhanced MRI (%)	Joint diagnosis (%)
Sensitivity	72.44	75.86	80.21
Specificity	81.56	83.73	89.11
Accuracy	93.78	78.62	88.82

**Table 3:** Pearson correlation coefficient test.

Index	CEUS vs. MRI	CEUS vs. CEUS + enhanced MRI	MRI vs. CEUS + MRI enhanced
Sensitivity	0.794	0.021	0.027
Specificity	0.063	0.128	0.003
Accuracy	0.102	0.389	0.173

The article "Contrast-Enhanced Ultrasound and Magnetic Resonance Enhancement Based on Machine Learning in Cancer Diagnosis in the Context of the Internet of Things Medical System" was retracted in 2023. Reasons: suspected computer-generated content; unreliable results or conclusions; lack of ethics approval or compliance; missing or withdrawn patient consent.

## Data Availability

The data underlying the results presented in the study are available within the manuscript.
